# IntOPMICM: Intelligent Medical Image Size Reduction Model

**DOI:** 10.1155/2022/5171016

**Published:** 2022-02-25

**Authors:** Piyush Kumar Pareek, Chethana Sridhar, R. Kalidoss, Muhammad Aslam, Manish Maheshwari, Prashant Kumar Shukla, Stephen Jeswinde Nuagah

**Affiliations:** ^1^Department of Computer Science Engineering & Head IPR Cell, Nitte Meenakshi Institute of Technology, Bangalore, Karnataka, India; ^2^Department of Computer Applications, Sivananda Sarma Memorial R.V. College, Bangalore, Karnataka, India; ^3^Sri Sivasubramaniya Nadar College of Engineering, Chennai, India; ^4^Department of Mathematics, College of Science, King Khalid University, Abha, Saudi Arabia; ^5^Department of Computer Science and Applications, MCNUJC, Bhopal, Madhya Pradesh, India; ^6^Department of Computer Science and Engineering, Koneru Lakshmaiah Education Foundation, Vaddeswaram, Guntur 522502, Andhra Pradesh, India; ^7^Department of Electrical Engineering, Tamale Technical University, Tamale, Ghana

## Abstract

Due to the increasing number of medical imaging images being utilized for the diagnosis and treatment of diseases, lossy or improper image compression has become more prevalent in recent years. The compression ratio and image quality, which are commonly quantified by PSNR values, are used to evaluate the performance of the lossy compression algorithm. This article introduces the IntOPMICM technique, a new image compression scheme that combines GenPSO and VQ. A combination of fragments and genetic algorithms was used to create the codebook. PSNR, MSE, SSIM, NMSE, SNR, and CR indicators were used to test the suggested technique using real-time medical imaging. The suggested IntOPMICM approach produces higher PSNR SSIM values for a given compression ratio than existing methods, according to experimental data. Furthermore, for a given compression ratio, the suggested IntOPMICM approach produces lower MSE, RMSE, and SNR values than existing methods.

## 1. Introduction

Through telemedicine, patients can receive medical care even if they are in a remote location. This technology allows remote patients to communicate with local hospitals and receive treatment without leaving their home [1]. However, storing and transferring large amounts of photographs in a hospital consume a large amount of bandwidth [2, 3]. To remedy the difficulty described above, compression is recommended. Images are compressed using a lossless compression approach in medical applications such as X-rays and X-ray images, because every information is vital [4]. In other words, loss compression techniques are used to compress the DC or video image. Wavelet transform is a highly efficient technique for decoding and encoding techniques such as cosine transform that delivers superior results but handles data in a serial way, requiring more processing time. Lossy compression is recommended for artificial neural networks to overcome these flaws [5]. A “bottleneck” network is one that has a big input layer that feeds into a small hidden layer, which is then merged into a huge output layer [6]. The bottleneck artificial neural network is a new image converter that analyses data continuously, using less time and thus being more efficient than other methods.  Figure 1 shows the bottleneck artificial neural network's topology.

Through telemedicine, patients can receive medical care even if they are in a remote location. This technology allows remote patients to communicate with local hospitals and receive treatment without leaving their home [7]. However, storing and transferring large amounts of photographs in a hospital consume a large amount of bandwidth [8]. Through telemedicine, patients can receive medical attention even if they are in a remote location. However, unlike in traditional hospitals, medical images are often large and require a large amount of bandwidth to store and transmit [9].

The outcome of the concealed layer, on the other hand, is a decimal value between 1 and 1. This indicates that if we combine another compression technique with the output of the hidden layer, we can compress it even more. As a result, the codebook in this study was developed using the new GenPSO hybrid approach [10]. The codebook is then utilized to condense the hidden neurons as a vector volume. Because of its capacity to process preimplant models to build simpler models with fewer components, this artificial neural network is better suited for picture reduction [11]. It offers the benefits of a simple structure, stability, and easy hardware performance, but its network training issues are related to large-scale optimization, which affects algorithm specificity over time due to its drawbacks: long duration and a low starting price. To address this disadvantage, an optimization strategy is required. As a result, the network is optimized using a GenPSO hybrid approach in this article [12].  Figure 2 depicts our proposed blockbuster neural network design for image compression.

The following are the primary contributions of this study.

To compress medical images, a bottleneck type artificial neural network was designed.

- GenPSO, a novel hybridized approach for optimizing neural network parameters, is developed
- The hidden layer of a bottleneck type artificial neural network is compressed more effectively with GenPSO, resulting in a higher compression ratio
- A high compression ratio and superior performance over existing methods are achieved
- For a real-time medical data set, the proposed technique produces good results

This document's manuscript is arranged as follows: The second section looks at some recent literature that is pertinent. The suggested architecture is described in depth in Section 3. The experimental results are shown in Section 4, which comprise general operational results of comparing the performance of GenPSO and other compression methods previously reported.  Section 5 contains the conclusion and recommendations for future work.

## 2. Background

Various traditional approaches such as JPEG [9], JPEG 2000 [10], SPHIT [11], EBCOT [12], and lifting scheme [13] have been developed for medical image compression, as well as current approaches such as artificial intelligence-based approaches such as neural network-based approaches. Artificial intelligence-based technologies are found to be superior to traditional approaches when dealing with incomplete or noisy data. These methods are not only computationally efficient, but they are also near-perfect in terms of decision-making accuracy. The authors of [14] proposed a neural network-based technique based on edge preservation. In this network, quantization levels were used to represent compressed patterns, and the compression ratio was determined by computing the average mean square value. The authors of [15] proposed a neural network with vector quantization that created a set of codes using the self-organizing feature map algorithm. As a result, all of the blocks created by each code vector were then modelled using a cubic surface to provide a built image with significant perceptual fidelity. The authors presented a multi-resolution-based neural network compression technique in [16], which was well suited to low bit rate coding with coarsely quantized digital coefficients. With the use of reference coefficients, a filter bank was also used to accurately synthesize the signal. This method was superior to conventional methods only for low bit rate compression; however, at high bit rates, its performance deteriorated dramatically. The authors of [17] presented a DCT-based neural network compression approach. To associate the grey image intensity, i.e., pixel value during compression, DCT coefficients were employed in conjunction with a neural network based on supervised learning, which was generally trained with a single ideal compression ratio. The authors reported a lossless compression solution for medical pictures using a neural network and an enhanced back-propagation algorithm in [18], which demonstrated significant compression performance but only with low PSNR. The authors of [19] proposed a medical compression algorithm that included a neural network and a Haar wavelet with nine compression ratios. The main drawback of this technique was that the compressed image quality was poor, making it unsuitable for medical image processing. The authors of [20] proposed an image compression technique for medical images that used wavelet and radial basis function neural network (RBFFN) features, as well as vector quantization. The medical images were decomposed at different resolutions with distinct frequency bands and then compressed using wavelet filters to create a set of sub-bands. Then, based on their statistical features, several quantization and coding procedures were used. RBFFN was used to compress the high-frequency coefficients, whereas differential pulse code modulation (DPCM) was used to compress the low-frequency band coefficients. In addition, the RBFFN hidden layer coefficients were vector quantized to increase the compression ratio without damaging the reconstructed image. The authors of [21] proposed a compression method based on artificial neural networks. The image content was included in the compression process, resulting in dramatically enhanced compression quality. An upstream module grouped the appearing image contents and identified the compressor using the unsupervised trained artificial neural network. The compressors utilized in this approach were then set up as artificial neural networks that had been trained using supervised learning and evolved into specialists for certain image contents during their training. A dataset is a collection of all these subset photographs of a single image that is normally partitioned into a number of images. Our dataset also contains similarity of specific image contents, which is thoroughly utilized by this proposed approach. As a result, this compression technique provided superior compression performance and image quality when reconstructed. The dual-level DPCM, which consisted of a linear DPCM followed by a nonlinear DPCM known as context-adaptive switching neural network (CAS-NNP), was presented as a lossless compression method for medical photographs in [22]. Based on the context texture information of the predicted pixel present in the image, this CAS-NNP was frequently switched between three neural network predictors. As a result, this strategy resulted in a smaller prediction error. For compression, the authors suggested a hybrid predictive wavelet coding with neural network in [23]. Inter-pixel redundancy was reduced by applying predictive coding to preprocess the image data values, and then discrete wavelet transforms the difference calculated between anticipated and original values, known as an error. The properties of both predictive and discrete wavelet coding were combined in this way. The nonlinear neural network predictor used the predictive coding procedure in this case. As a result, as compared to JPEG 2000, this compression approach produced higher-quality compressed images at high decomposition levels. The authors of [24] suggested an image compression technique based on artificial neural networks, in which the original image was coded in terms of both pixel coordinates and pixel values. To do so, the image was first read as a matrix with dimensions *m* ∗ *n*, and then, a pair of pixel values and counts was created by searching for co-similar pixel coefficients. For the obtained co-similar pairs, the suggested procedure is quite similar to the run-length encoding technique. These pairs were then sent into a neural network, which was used to compress the image losslessly. The authors of [25] proposed an image compression approach in which the images were digitized first and then wavelet transforms were applied. The result, i.e., transformation coefficients, was then vector quantized to the nearest integer values. Following quantization, the coefficients were encoded using the Huffman encoding, which compressed the tablet images and the tablet strip images derived from the text's exact frequencies. As a result, a variable length code table was created, with source symbols encoded, stored, and then sent via the channel for decoding. Unsupervised neural networks were used to improve image quality and remove block artefacts in this case. The authors of [26] suggested a medical image compression method based on the radial basis function of a neural network. The neural network had two layers of feed-forward network, with hidden nodes implemented using a series of radial basis functions and output nodes implemented using linear summation functions, similar to multilayer perceptron (MLP). The entire network training was broken into two sections here. The weights from the input layer to the hidden layers were determined in the first stage, and the weights from the hidden layer to the output layer were determined in the second stage. Additionally, the neurons were added to the network's hidden layer until the MSE target was met. The network that was created here was excellent at interpolation. Approximating functions can also be done with the radial basis network. The authors of [27] presented a compression method based on the back propagation of discrete wavelet transform-fed neural networks. The photographs were initially compressed using the DWT technique, and then, the images from the DWT step were fed into a back-propagation neural network for additional compression. The PSNR value and compression ratio of the final compressed image were both improved. The authors introduced a deep neural network (DNN) compression approach based on rectified linear units (ReLUs) in [28]. The capabilities of DNNs were used in this technique to find a substantial estimate of the link between compression and decompression. The ReLUs speed up the encoding and decoding processes, increased the DNN's ability to generalize, established efficient gradient propagation, induced sparsity, and made it computationally efficient. As a result, ReLUs improved the ability of these neural networks to conduct real-time compression. The authors of [28] proposed a compression strategy based on a feed-forward neural network. Image quality was kept via predictive image coding. The medical image was first partitioned into diagnostically important regions (DIRs) and non-DIRs using a graph-based segmentation strategy in this method. The prediction step was then carried out using identical feed-forward neural networks (FFNNs) at both the compression and decompression stages. The gravitational search method and particle swarm techniques were used to train FFNNs. Then, using lossless and near-lossless mannered methods, the performance of these two FFNNs was assessed. This prediction error sequence was further reduced using the Markov model-based arithmetic coding to calculate the difference between actual and predicted pixel values.

## 3. Materials and Methods

The following is the image compression technique utilizing our GenPSO technology. In our work, we use vector quantization for image compression. The picture pixel is encoded using the codebook approach by vector quantization. Creating a codebook can be thought of as a search issue, with the goal of finding the best solution, since the representative codebook can be used to compress images properly. To clone VQ, we must meet the following two requirements: 1. the method used to create the greatest laptop, and the job's algorithms are listed below; and 2. codebook standards that are the most representative. As a result, a new generation of GenPSO will be employed to conduct the search for the optimal codecs. The grey scales represent the source of the training model inside the scientific framework. That is, the image will be chopped into identical-sized blocks as the training model. The training sample will be used to pick the majority of avatars. The representative photographs will be punished and categorized in the codebook according to the categorization and selection procedure. These procedures are followed to make a codec with GenPSO: the GenPSO structure uses a method of encoding real numbers and sticks to chromosomal codes as a single solution. It also generates the first population based on the picture block's vector training. Calculating the GenPSO evolution shows that the original population is a viable answer. In this study, we employ the crossover selection operator and the exchange operation to produce the best logic codebook using the PSNR as a fitness value lower than the measurable threshold. The process for optimizing the parameter network using our GenPSO method is as follows. The GA solution determines the starting population of PSO in our hybrid approach to GA and PSO. GA and PSO evenly dispersed the number of repetitions. The GA governs the first half of the exchange, and the solution is supplied as the first set of PSOs. PSO owns the remainder of the exchange. As a result, it can solve the problem of sluggish network convergence and reduce BP algorithm recurrence. Both global and local hybrid searches should be included in the suggested strategy. After that, for each particle, the optimal Pg positions are constructed, which are subsequently assigned to the BP algorithm to refine these search operations.

The first step in the process is to determine the starting population of PSO in the hybrid approach to maximize the efficiency of the parameter network. The solution is then divided into two groups, namely the first group of PSOs and the second group of PSOs.

### 3.1. Artificial Neural Network

The image compression problem is solved using the neural network architecture depicted in Figure 3. The input from a high number of input neurons is sent to a smaller number of neurons in the hidden layer, which are then provided to a larger number of neurons in the network's output layer. The forward neural network for communication is the name for this type of network.

The network's architecture consists of 64 hidden neurons and 16 output neurons. The encoded information collected by the hidden layer's neuron is sent to the encryption layer, which then decodes it. The resulting output layer is composed of 16 hidden nodes.

To control the output of the hidden layer, we need to combine the output with other compression techniques. This method is proposed as a hybrid approach that combines neural networks and GenPSO.

### 3.2. Updation of Weights in Neural Network Using GenPSO

The weight generated by the neural network is updated using the GenPSO algorithm in this stage. A chromosome's initial constitutive population has an evenly distributed random number. The weight of the neural network is represented by the chromosome. A crossover on a node is what we are talking about here. Two springings are created from the parent, each active node from a hidden layer and several outputs, all of which are randomly chosen with equal chance. This node is referred to as a transit node. With the other master, the value of all input weights for that particular node is altered. This update can alternatively be thought of as a node change, with all incoming weights for randomly chosen active nodes. Finally, the PSO method is used. A GA decision was used to establish the initial PSO population. As a result, it can solve the GPS network's sluggish convergence problem.

#### 3.2.1. Algorithm for Weight Evolution by GenPSO in ANN

To get the best weight value, the following procedures are examined:

- On area *M* is *R*_*n*_, the population of the XiMi a solution, *I* = 1,…, is began.
- Using a parent population distribution, two parents are chosen at random, and two births are generated using a crossover operator.
- The offspring are subjected to hereditary mutation.
- Step (ii) is repeated until the number of offspring *o* is equal to the number of parents. Otherwise, Step 2 is proceeded.
- In light of the objective function, any parental decision, *I* = 1,…, and progeny *X*o, *o* = 1,…, are estimated (*X*).
- Mixed population *X*_*m*_, *m* = 1,…, 2, Both the parent population and the population formed. This mix is randomly mixed so that parents and children mix up properly.
- Each *X*_*m*_, *m* = 1,…, 2 answer is compared to 10% of the solutions of the other randomly selected solutions from a mixed population.
- The decision on the highest wages is left to the next generation of parents.
- If the best chromosome difference across *N* generations is less than the given brightness, the latest generation's best chromosome is the optimum weight; otherwise, the next step (ii) is proceeded.
- The genetic algorithm determines the initial particle population, as well as their location and velocity.
- The fitness value of all particles based on the fitness function and the optimization problem's aim is estimated.
- The values of each particle's fit are compared with its holes. The current fitness value is set to its pbest if the current value is better than pbest. Otherwise, the pbest value will remain unchanged.
- The population's current best fitness value is determined from all fitness values. Then, this value is compared to Gebel, and if it is better than Gebet, the current value is set to Gebel; otherwise, blank is left.
- Each piece's position and speed should be updated.
- If the best solution is identified that fits the predetermined minimum error or reaches the maximum number of repetitions, then the step is stop; otherwise, steps (*x*) through (xv) are continued.

### 3.3. Training Algorithm for Feed-Forward Neural Network

The neural network retardation algorithm follows the following stages to achieve high picture compression and real-time image compression.

Step 1: first and foremost, weight is required to begin with small random numbers. The input signal is received by each input neuron, which then passes it to the hidden unit.
Step 2: weighted input signals from hidden neural network units are combined with the following spacing:
  (1) $$\begin{array}{c} z_{\text{inf}}=v_{oj}+\sum_{i=1}^{n}x_{i}v_{ji}. \end{array}$$
On application of activation function, the *z*_*j*_ = *f* (*z*_inf_) is output and it sends this signal to all neurons of the output layer.
Step 3: now, neurons (*y*_*k*_, *K*=1, .., *m*) are output, all weighted inputs *y*_*ink*_=*w*_*ok*_+∑_*j*=1_^*p*^*z*_*i*_*w*_*jk*_) are added and its activation function is applied to calculate the output:
  (2) $$\begin{array}{c} y_{k}=f\left(y_{ink}\right) \end{array}$$
Step 4: output unit compares the calculated output corresponding to a target, and error is calculated as follows:
  (3) $$\begin{array}{c} \sigma_{k}=\left(t_{k}-y_{k}\right)f\left(y_{ink}\right). \end{array}$$
Step 5: the error from the output is distributed to the hidden layer, and then, each hidden unit (*z*_*j*_, *j*=1,…, *n*), sums its inputs from units in the layer:
  (4) $$\begin{array}{c} \sigma_{inf}=\sum_{k=1}^{m}\delta_{j}w_{jk}. \end{array}$$
The error is calculated as follows: *σσ j* = in *f* (z). (7)
  (5) $$\begin{array}{c} \sigma_{j}=\sigma_{inj}f\left(z_{inj}\right). \end{array}$$
Step 6: each output neuron (*y*_*k*_) updates its bias and weights (*j* = 1,…,*p*), and the weights are corrected by
Δ*w*_*jk*_=*ασ*_*k*_*z*_*j*_, and similarly, the bias is corrected by the term Δ*w*_*jk*_=*ασ*_*k*_.
Step 7: the newly updated weights are represented by the following terms:
  (6) $$\begin{array}{c} w_{jk}\left(\text{updated}\right)=w_{jk}\left(\text{old}\right)+\Delta w_{jk},\\ w_{ok}\left(\text{updated}\right)=w_{ok}\left(\text{old}\right)+\Delta w_{ok}. \end{array}$$
Step 8: the weight correction term for hidden neurons is as follows:
  (7) $$\begin{array}{c} \Delta v_{ij}=\alpha \sigma_{j}x_{i}. \end{array}$$
The bias correction term for hidden neurons is as follows:
  (8) $$\begin{array}{c} \Delta v_{oj}=\alpha \sigma_{j}. \end{array}$$
Step 9: newly updated weights are as follows:
  (9) $$\begin{array}{c} v_{ij}\left(\text{updated}\right)=v_{ij}\left(\text{old}\right)+\Delta v_{ij},\\ v_{oj}\left(\text{updated}\right)=v_{oj}\left(\text{old}\right)+\Delta v_{oj}. \end{array}$$

Together with the GenPSO algorithm, forward back-propagation algorithms are used to train neural networks. Vector quantization techniques are used to increase the compression ratio.

### 3.4. Image Compression Using Vector Quantization

The construction of a codebook that maximizes PSNR while minimizing bit rate and computing time is a critical challenge with VQ picture compression. We will look at the factors that influence the VQ algorithm in this part. Code: a mapping from a vector to a k-measured Euclidean space (Rk) in a restricted set C containing a N output called code words is called a VQ of dimension *k* and size *N*. Q: Rk → C, where *C* = (*y*1, *y*2,…, *yN*), and yi ∈ Rk for each *i* ∈ J ≡ {1, 2 …, *N*}. The codebook is the set C. The vector volume solution is *r* = (log2N)/*k*, which measures the number of bits of vector components needed to represent the input vector and indicates whether the codec is well-designed. A 2 × 2 block is used to generate code words in a straightforward way. To achieve a lower bit rate, we must either raise the *k* size or the block size. Large block size, on the other hand, will result in reduced PSNR because the coding data are generated by the block's optimal pixel intensity. In contrast, reducing the block size improves the PSNR because small block coding absorbs the difference between the intensity value and the block size. A high bit rate is advantageous in this instance. We suggest a VQ picture encoding that boosts PSNR while maintaining the same bit rate in this study. To achieve these conditions, the first codebook must be created using an optimization technique.

### 3.5. Using the GenPSO Vector Quantization Approach to Compress Images

The picture pixel is encoded using the codebook approach by vector quantization. Creating a codebook can be thought of as a search issue, with the goal of finding the best solution, since the representative codebook can be used to compress images properly. To clone VQ, we must meet the following two requirements: 1. the method used to create the greatest laptop, and the job's algorithms are listed below; and 2. codebook standards that are the most representative. As a result, a new generation of GenPSO will be employed to conduct the search for the optimal codecs. The image is divided into 4 × 4 pixel pieces during digital code production. These blocks are transformed into e-dimensional vectors, which are referred to as training vectors, and the collection of training vectors is referred to as a vector training set of size N [8]. The equation is used to determine N.

(10) $$\begin{array}{c} N\;=\;\frac{\left(m\times m\right)}{k}, \end{array}$$

where *k* is the vector size and *m* × *m* is the number of rows and columns of pixels in the input image. The p location for which the encoder is to be selected is calculated using the following equation:

(11) $$\begin{array}{c} p\;=\;\frac{N}{M}, \end{array}$$

where *N* is the size of the training set and *M* is the desired size of the codebook. The coders at each location of the training set were selected to form the coding book.

In the coding step, the nearest coders for each training vector were determined by calculating the distance *d* (*e*, *c*) using the following equation.

(12) $$\begin{array}{c} d\left(Y,X_{i}\right)=\sum_{j=1}^{16}\left(y_{j}-x_{ij}\right). \end{array}$$

There must be a minimum for I *j* where *I* = 1 to *M* and *d* (*Y*, *X*_*i*_). Each block of the input image is replaced with the converter's index, which corresponds to (3). Index cards are a collection of such indicators. Now, the compressed image is stored or supplied as a map index and code. Each index in the index code is replaced by the correct encoder at the decoder step, when you regenerate the image from the compressed image. The initial codebook in the proposed GenPSOVQ technique is generated by the GenPSO algorithm. The procedure for determining the best codebook is as follows:

- On area *M* is *R* n, the population of the XiMi a solution, *I* = 1,..., is began.
- Using a parent population distribution, two parents are chosen at random, and two births are generated using a crossover operator.
- The offspring are subjected to hereditary mutation.
- Step (ii) is repeated until the number of offspring *o* is equal to the number of parents. Otherwise, Step 2 is proceeded.
- In light of the objective function, any parental decision, *I* = 1,…, and progeny *X*o, *o* = 1,…, are estimated (*X*).
- Population mix *X*_*m*_, *m* = 1,…, 2. The initial population, as well as the new one, was born out of the original population. This mixture is mixed at random to ensure that parents and children are suitably mingled.
- Each *X*_*m*_, *m* = 1,…, 2 answer is compared to 10% of the solutions of the other randomly selected solutions from a mixed population.
- The decision on the highest wages is left to the next generation of parents.
- If the best chromosome difference across N generations is less than the given brightness, the latest generation's best chromosome is the optimum weight; otherwise, the next step is proceeded.
- The genetic algorithm determines the initial particle population, as well as their location and velocity.
- The fitness value of all particles based on the fitness function and the optimization problem's aim is estimated.
- The values of each particle's fit with its holes are compared. The current fitness value is set to its pbest if the current value is better than pbest. Otherwise, the pbest value will remain unchanged.
- The population's current best fitness value is determined from all fitness values. Then, this value is compared to Gebel, and if it is better than Gebet, the current value is set to Gebel; otherwise, blank is left.
- The pace and position of each item are adjusted.
- If the best solution is identified that fits the predetermined minimum error or reaches the maximum number of repetitions, then the step is stopped; otherwise, steps (*x*) through (xv) are continued.

### 3.6. Proposed Image Compression Using GenPSO Vector Quantization Neural Network Approach

The following steps explain the suggested technique for quantifying vectors using reverse neural networks:

  Step 1: the image is cut into eight separate sections. These cartridges have a square shape to them. A symmetric matrix is simple to work with.
  Step 2: the matrix's pixel value (0 to 255) is determined.
  Step 3: these values are applied to the forward neural network. Because the detector is 8 by 8, this network must contain 64 input nodes. The training algorithm described in Section 3 is used to train the neural network.
  Step 4: GPS-added weight and tilt are sent into a hidden layer with 2, 4, 8, 16, 32, and 64 hidden nodes. As described in Section 3.4, these values are encoded using GenPSOVQ.
   Step 5: after completing the training, the 8 × 8 printer is selected in the correct order.
  Step 6: digital bits are turned into real numbers.
  Step 7: finally, at the output of the nervous system's output layer, the call phase displays depressed images (output images). During the compression and decompression process, a pixel is converted to a true value and a true value is converted to a pixel.

## 4. Experimental Results

### 4.1. Dataset Used

PSNR, MSE, SSIM, NMSE, SNR, and CR [28] values are used to assess the performance of the proposed IntOPMICM approach on real-time medical pictures. These findings are compared to those of known algorithms such as FFNN, VQFFNN, optimized FFNN, and optimized VQFFNN.  Figure 4 shows a selection of photographs from a real-time medical database [29].

### 4.2. Performance Metric

For the assessment of the compression approaches, this study employs six metrics namely PSNR, MSE, SSIM, NMSE, SNR, and CR.

#### 4.2.1. Peak Signal-to-Noise Ratio

To compare the quality of the compressed and original images, the peak signal-to-noise ratio (PSNR) is utilized. The formula for PSNR is as follows:

(13) $$\begin{array}{c} \text{PSNR}=10\times \;\log10\frac{255\times 255}{1/\text{H}\times \text{W}\sum_{x=0}^{H-1}\sum_{y=0}^{W-1}{\left[f\left(x,y\right)-g\left(x,y\right)\right]}^{2}}\text{dB,} \end{array}$$

where *H* and *W* are the image's height and width, respectively, and *f*(*x*, *y*) and *g*(*x*, *y*) are the grey levels in the original and compressed images, respectively, at coordinates (*x*, *y*).

#### 4.2.2. Structural Similarity Index

The structural similarity index is a means of determining how similar the compressed and original images are.

(14) $$\begin{array}{c} SSIM\;\left(y,\;\hat{y}\right)=\;\frac{\left(2_{\mu_{y}\mu_{\hat{y}}}+\;c_{1}\right)\left(2\sigma_{y\hat{y}}+\;c_{2}\right)}{\left(\mu_{y}^{2}+\;\mu_{\hat{y}}^{2}+\;c_{1}\right)\left(\sigma_{y}^{2}+\;\sigma_{\hat{y}}^{2}+\;c_{2}\right)}, \end{array}$$

where $\hat{Y}$ is the compressed image, the *Y* is the original image, µ is the mean, and σ2 is the variance.

#### 4.2.3. Mean Square Error

The difference between a compressed image [30] and the original image is measured using the mean square error (MSE). The MSE can be calculated using the following formula:

(15) $$\begin{array}{c} MSE=\;\frac{1}{n}{\sum_{i=1}^{n}\left({\hat{Y}}_{i}-\;Y_{i}\right)}^{2}, \end{array}$$

where $\hat{Y}$ is the compressed image and the Y is the original image.

#### 4.2.4. Root-Mean-Square Error

The root-mean-square error (RMSE) is a frequently used measure of the difference between compressed image values and original image values.

(16) $$\begin{array}{c} RMSE=\;\sqrt{\frac{\sum_{i=1}^{n}{\left({\hat{Y}}_{i}-\;Y_{\;i}\right)}^{2}}{n}}, \end{array}$$

where $\hat{Y}$ is compressed image and Y is the original image.

### 4.3. Experimental Analysis

#### 4.3.1. Experiment No. 1: Analysis of Proposed IntOPMICM Compression Approach

We will evaluate the contribution of the suggested IntOPMICM compression technique in this experiment. The PSNR, MSE, SSIM, NMSE, SNR, and SNR versus a 25% CR ratio are used to assess the scheme's performance. It is depicted in equations (4)–(7), respectively. The PSNR, MSE, SSIM, NMSE, SNR, and SNR measurements of IntOPMICM, as well as the current techniques, are listed in Table 1 and depicted in Figure 5.

#### 4.3.2. Experiment No. 2: Performance of Best Chromosome Particles of GenPSO with 50 Population Size

The 2-2-1 feed-forward architecture was designed, and the error value is evolved according to the GenPSO method set out above. The population size is 50, and the termination rule is if the best error in the chromosome in the 50 successive generations is less than 0.00001, as shown in Figure 6.

#### 4.3.3. Experiment No. 3: Performance of Best Chromosome Particles of GenPSO with 100 Population Size

The architecture of the best chromosome particle distribution 2–2–1 was developed using the GenPSO method described above. The population size is 50, and the termination rule is if the best error in the chromosome in the 50 successive generations is less than 0.00001, as shown in Figure 7.

#### 4.3.4. Experiment No. 4: Performance of Error of GenPSO with 50 Population Size

The 2-2-1 feed-forward architecture was designed, and the error value is evolved according to the GenPSO method set out above. The population size is 50, and the termination rule is if the best error in the chromosome in the 50 successive generations is less than 0.00001, as shown in Figure 8.

## 5. Conclusion

Image-based processing is becoming increasingly used in a variety of applications. There are numerous approaches that give satisfying results to some extent. However, with evolving technology, there is still a lot of room for growth in this field. The IntOPMICM approach, which combines GenPSO and VQ, has been introduced as a novel image compression scheme. A combination of fragments and genetic algorithms was used to create the codebook. PSNR, MSE, SSIM, RMSE, SNR, and CR indicators were used to test the suggested technique using real-time medical imaging. The suggested IntOPMICM approach produces higher PSNR SSIMM values for a given compression ratio than existing methods, according to experimental data. Furthermore, for a given compression ratio, the suggested IntOPMICM approach produces lower MSE, RMSE, and SNR values than existing methods. Various image-based processing techniques are becoming increasingly popular in various applications. IntOPMICM, which combines VQ and GenPSO, is a novel algorithm that combines genetic algorithms and fragments. It was tested using real-time medical images.

## Figures and Tables

**Figure 1:** Structure of the bottleneck artificial neural network.

**Figure 2:** Proposed blockbuster neural network architecture for image compression.

**Figure 3:** Bottleneck type feed-forward neural network.

**Figure 4:** Experimental images.

**Figure 5:** Analysis of PSNR, MSE, SSIM, NMSE, and SNR of IntOPMICM approach along with 25% CR ratio.

**Figure 6:** Performance of best chromosome particles of GenPSO with 50 population size.

**Figure 7:** Performance of best chromosome particles of GenPSO with 100 population size.

**Figure 8:** Performance of error of GenPSO with 50 population size.

**Table 1:** Analysis of PSNR, MSE, SSIM, NMSE, and SNR of IntOPMICM approach along with 25% CR ratio.

Dataset					
Compression approaches					
Metrics	FFNN	OFFNN	VQFFNN	VQOFFNN	IntOPMICM
PSNR	35.6556	36.8041	48.1246	49.6515	52.4227
SSIM	0.0120	0.2053	0.4327	0.5323	0.1736
MSE	17.6814	13.5729	8.8603	6.1953	1.4164
RMSE	4.2049	3.6841	0.0011	2.4890	1.1901
SNR	25.5966	21.4276	16.9645	10.6537	7.4263

## Data Availability

The data that support the findings of this study are available on request from the corresponding author.
